RETRACTED

# Fabrication of an Ocular Prosthesis for a Pediatric Retinoblastoma Patient by a Simplified Technique

**DOI:** 10.5005/jp-journals-10005-1061

**Published:** 2010-08-17

**Authors:** Arpan Pavaiya, Vikram Saumyendra Singh, Pooran Chand, Dayal Raghuvar Singh

**Affiliations:** 1 Department of Prosthodontics, Faculty of Dental Sciences, CSM Medical University, Lucknow, Uttar Pradesh, India; 2 Assistant Professor, Department of Prosthodontics, Faculty of Dental Sciences, CSM Medical University, Lucknow, Uttar Pradesh, India; 3 Assistant Professor and Head, Department of Prosthodontics, Faculty of Dental Sciences, CSM Medical University, Lucknow Uttar Pradesh, India

**Keywords:** Retinoblastma, enucleation, precooperative, ocular prosthesis.

## Abstract

Retinoblastoma is one of the more highly invasive and common intraocular malignancies of childhood. Treatment in most of the cases consists of enucleation followed by placement of orbital implants. Prosthetic rehabilitation is especially challenging in younger and precooperative pediatric patients. The following case report describes the rehabilitation of a 4-year-old child with retinoblastoma, with an ocular prosthesis fabricated by a simplified technique.

## INTRODUCTION

Surgical procedures in the removal of an eye can be broadly classified as–evisceration where the contents of the globe are removed leaving the sclera intact, enucleation (most common) where the entire eyeball is removed after severing the muscles and the optic nerve and exenteration where the entire contents of the orbit including the eyelids and the surrounding tissues are removed.^1^

Enucleation in early childhood hinders normal growth process and if the etiology was malignancy, the accompanying radiation treatment further retards development. For psychological, social and esthetic reasons ocular prosthesis should be fabricated as early in life as possible.^2^ To prevent the orbit from shrinking and to promote development of lids and lining soft tissues, a prosthesis of a larger size must be fabricated from time to time as the child grows.^3^ The socket is fully developed at about twelve years of age, from when the teenage patients should be treated as adults.^1^

## CASE REPORT

The patient was a male child of 4 years, who reported to the Department of Ophthalmology with complaints of whitish spot on the right eye accompanied by bulging and squint, and pain on movements as narrated by his father. He was diagnosed with retinoblastoma and the enucleation was performed immediately. An orbital implant was not planned at the time of the surgery as regular periodic examinations were planned to rule out any recurrences at the optic nerve head, and placement of an implant could hinder early clinical and radiological detection. The patient was then referred to the Department of Prosthodontics for the fabrication of prosthesis (Fig. 1).

RETRACTED

After examination and working out of treatment protocol, the work plan explained to the patient by simple diagrams and posters to gain his cooperation.^4^ The procedure was initiated by selecting and modifying a prefabricated (stock) eye whose iris and pupil closely matched that of the natural eye, to comfortably and loosely fit the socket. This was duplicated with clear heat cured PMMA (Trevalon, Dentsply India Pvt. Ltd., Gurgaon, India) and perforated for use as a tray in the impression procedure. Perforation of the tray was done to avoid any compression of the ocular tissues. The tray was placed in the socket and the patient was asked to gaze at a distant point to accurately mark the pupil as per contralateral side, on the tray.

A thin tube (1 mm diameter, 2 cm length) was fabricated to serve as a handle for the impression tray and attached at the pupillary point for proper tray orientation during impression making (Fig. 2). A thin mix of ophthalmic alginate (Ophhal-mic moldite, Milton Roy Co. Sarasota Fla.) was then injected in the socket and loaded on the tray which was placed into the position. The child was asked to make all eye movements to allow the alginate to flow into all extensions as well as onto the tray’s outer surface to record lid movements, while taking care that the tray handle replicated the pupillary position of the natural eye. Impression was examined for accuracy (Fig. 3) and the cast was poured in two seperable parts with 2nd part being poured after applying lubricant and making orientation grooves on the first half after it had partially set (Fig. 4). The tube was maintained as a sprue to pour the wax pattern and to transfer the pupillary point onto the cast.

The technique was modified here by orienting the previously mentioned stock eye on the cast according to previously transferred pupillary mark. Liquified modeling wax was then poured into the cast and the stock eye was positioned in its previously oriented position, in the wax pattern. This stock eye-wax pattern combination was tested in the socket and modified for adequacy of ocular movements, correction of pupillary alignment, proper palpebral movements, scleral contour and convexity of the left eye. The next step was to reproduce scleral shade of the left eye. For this, shade tabs were prepared by mixing and matching different shades and proportions of tooth colored acrylic till the color of sclera of the other eye was replicated. Then the adjusted and modified stock eye-wax pattern combination was invested, flasked and dewaxing was done. Red silk fibers to mimic veins were placed in the dough of the predeter-mined acrylic shade followed by routine curing, finishing and polishing. Finally a thin film of the sclera was removed and replaced by a clear film of transparent heat cured PMMA (Trevalon, Dentsply India Pvt. Ltd., Gurgaon, India) to copy corneal translucency. The properly finished and polished prosthesis was inserted in the socket after being disinfected and lubricated with an ophthalmic lubricant (Ecotears)^5^ (to maintain a tear film over the prosthesis and to improve eye movements). Minor adjustments were made at the time of delivery as per the patient’s comfort and esthetics (Fig. 5). Necessary instructions for cleaning, placing and taking out of the prosthesis were given and the need for regular recall appointments was emphasized.

RETRACTED

**Fig. 1:** Preoperative view

**Fig. 2:** Impression tray with tube in place

**Fig. 3:** Impression in alginate

**Fig. 4:** Cast poured in two portions with pupillary portion marked

**Fig. 5:** Postoperative view

## DISCUSSION

Anophthalmos is a condition in which no eyeball can be found in the orbit.^6^ Trauma is the most common cause for removal of an eye. The other common causes being glaucoma, malignancy, congenital deformities and infection. Retinoblastoma is the most common primary intraocular malignancy of the children which arises from immature retinal cells in one or both eyes between the ages of 6 months to 5 years equally in all races and both genders.^7^ Surgical removal of eye is the management in majority of the patients with unilateral retinoblastoma involving more than half the retina, though the induction of chemotherapy has modified this approach in many cases.^8^

Two options are available for artificial eye prosthesis, one is a prefabricated ocular prosthesis and other is custom made. Prefabricated eye prosthesis carry disadvantages of poor fit (which endangers the eye to granuloma formation), poor esthetics and poor eye movements. Custom made prosthetic eye fabrication involves complex painting procedures in various stages which are quite difficult and based purely on painting skills of the operator. The techinique to fabricate ocular prosthesis in this case report modifies a prefabricated eye prosthesis to a custom made fit and esthetics. This helped us to overcome the disadvantages of poor fit and esthetics of prefabricated prosthesis and complex painting procedure involved in making a custom made ocular prosthesis.

The purpose of this case report is to document a simpler technique for the fabrication of ocular prosthesis which does not depend much on artistic ability of the operator and is relatively easy to be performed by a dentist along with saving on laboratory time. The close adaptation of the custom made ocular prosthesis to the tissue bed provides maximum comfort and restores full physiologic function to the accessory organs of the eye.^3^ Voids that collect mucus and debris, which can irritate the mucosa and act as a potential source of infection may also be minimized and this prosthesis also provides optimum cosmetic and functional results.^3^

RETRACTED

Limitations of this technique are that the clinician has to depend on the availability of properly matching iris and pupillary part in the prefabricated eyes available and the long-term color stability of the heat cured acrylic and its union with the stock eye will have to be monitored.
